# The Collection and Recognition Method of Music and Dance Movement Based on Intelligent Sensor

**DOI:** 10.1155/2022/2654892

**Published:** 2022-06-03

**Authors:** Jun Geng

**Affiliations:** School of Art, Shandong University of Finance and Economics, Jinan 250014, China

## Abstract

With the popularization and development of Internet of Things technology, a large number of music and dance videos have emerged in all walks of life. In this information age, video communication has become a widespread communication method. In the current music and dance collection process, most of the action frame information of the dance video is repeated, and the stage background and costumes of the dance action are too many to fully express the human body movement information. Based on these problems, this article will realize the application of the intelligent sensor-based action recognition technology in the field of dance movement collection and complete the collection and recognition of music and dance movements. The research results of the article show that: (1) in the dance video image extraction process, the feature recognition effect of the proposed algorithm is the highest among the three models. The recognition effect of the upper body is 66.1, and the recognition effect of the lower body is 61.0. The image recognition effect can reach 73.4. During the statistical experiments on the recognition of different regions of the human body, the recognition effect of the intelligent sensor model proposed in the article is still the highest among the three models. The recognition effect of the upper body is 33.9, and the recognition effect of the lower body is 33.9. The recognition effect is 34.5, and the recognition effect of the whole body is 40.7. (2) In the traditional music and dance collection mode, the *P* values of the four test parts are all greater than 0.05, indicating that in the traditional music and dance collection mode, the differences between the four test modules are not significant. Combined with the evaluation results of the three groups in the traditional music and dance collection mode, we can conclude that under the condition that the initial conditions are basically the same, and the training conditions and environment are basically the same, the trainees who use the smart sensor music and dance collection training method are better in physical fitness. The indicators have been better improved, and the effect is greatly optimized compared with the training effect in the traditional music and dance collection mode. (3) After the test set runs, the article proposes that the accuracy rate of the dance collection model based on the smart sensor algorithm is 88.24%, the accuracy rate can reach 88.96%, the improved accuracy rate can reach 91.46%, and the accuracy rate can reach 91.79%. The ROC curve value of the article and the improved model is very stable. The ROC value before the improvement remains at about 0.90, and the ROC value after the model improvement also remains at 0.96. After the test set runs, the performance of the four models has decreased to a certain extent, but the smart sensor dance acquisition model proposed in the article has the lowest degree of decline, and the performance after the decline is still the highest among the four models. The accuracy of the model is 90.24%, and the accuracy of the improved model is 93.16%. The ROC curve values of the improved system are very stable, the ROC value has been maintained at 0.95, and the ROC value before the improvement is stable within the range of 0.85–0.95. The experimental results further illustrate that the model proposed in the article has the best performance.

## 1. Introduction

Dance is a kind of traditional culture with the beauty and significance of movement. We must carry forward it. Dance is composed of many movements. One of the challenges of dance development is the effective connection between the movements. In recent years, music and dance video analysis has also become the research direction of many experts. Effective analysis of music and dance videos can not only correct dancers' posture, help dancers effectively train, but also play a certain role in the development of music and dance. *Promotion*. In view of the complexity in the dance learning process, the article decomposes complex dance videos into many small segments based on intelligent sensor technology, making the abstract content more intuitive and easy to understand. Reference [1] explored the way of perceiving the correspondence between music and body movement by analyzing the characteristic relationship between music and movement. Literature [2] studies collections with modern dance with the aim of providing libraries with an annotated bibliographic resource guide. Reference [3] proposed a gesture recognition algorithm for Indian classical dance style using Kinect sensor, which can achieve a high recognition rate of 86.8%. Reference [4] introduced the meaning of Laban movement analysis symbols and the method of dance movement recognition. Reference [5] proposes a gesture recognition implementation that uses hidden Markov models to classify specific gestures in traditional dance. Reference [6] proposed a fuzzy membership function to automatically recognize dance gestures. Reference [7] introduces the gesture recognition method and its application in the dance training system in the teaching virtual reality environment. Reference [8] applied the recognition of dance gestures to music performances, reversing the traditional music and dance interaction. Reference [9] builds a robust recognizer based on linguistic motivation method to recognize dance poses in Balinese traditional dance choreography. Reference [10] presents a complete manipulation prototype for compressing and recognizing dance gestures in contemporary ballet. Reference [11] presents an update of a project aimed at developing a modular system for real-time analysis of body movements and postures. Reference [12] proposes a tool for nonuniform subsampling of spatiotemporal signals with the goal of recognizing a set of dance gestures in contemporary ballet. In [13], an angle representation of the skeleton is designed for robustness under the noise input of the Kinect sensor. Reference [14] designed a 4-stage system for automatic gesture recognition in dance. Reference [15] proposed a new method for human gesture recognition based on quadratic curve, which achieved a recognition rate of up to 97.65% on a database of 16 different gestures.

## 2. Research on the Collection and Recognition Methods of Music and Dance Movements

### 2.1. Motion Capture Classification

After consulting relevant materials, we found out the common dance video capture systems. The details are shown in Table 1.

### 2.2. Design of Dance Gesture Capture

The research of this paper is based on the principle of intelligent sensor and applies motion capture technology to the process of dance pose extraction, so as to extract the skeleton movement route of the human body and establish a quantitative method for dance pose analysis. First, install data identification points on each part of the dance trainer's body, and then dance in a predetermined area, and the system will automatically capture the basic dance movements of the dancer. In this process, the system will match the collected dance movements with the dance movement database. When all the data collection points are successfully identified by the computer and entered into the system, the real-time collection of human dance movements has been successfully completed. The working roadmap of the scheme is shown in Figure 1.

## 3. Collection and Recognition of Music and Dance Movements by Smart Sensors

### 3.1. Dance Image Preprocessing

In this paper, the average value method is selected to grayscale the original image. This method obtains the gray value of the point by calculating the average value of the 3-channel brightness of each pixel point [18]. The corresponding mathematical expression is as follows:

(1) $$\begin{array}{c} \text{Gray}=\frac{\left(R+G+B\right)}{3}. \end{array}$$

Assuming that the value of a certain pixel of the video at time is *M*_*t*_, the random probability [19]is as follows:

(2) $$\begin{array}{c} P\left(M_{t}\right)=\sum_{i=1}^{k}\omega_{i,t}g\left(M_{t},\mu_{i,t},\sigma_{i,t}\right), \end{array}$$

where *K* is the number of Gaussian distributions, *ω*_*i*_ is the *i*-th Gaussian distribution weight, *μ*_*i*,*t*_ and *σ*_*i*,*t*_ represent the mean and variance, and *g* is the Gaussian distribution function.

(3) $$\begin{array}{c} \left|M_{t+1}-\mu_{i,t}\right|\leq 2.5\delta_{i,t}. \end{array}$$

Parameter update is as follows:

(4) $$\begin{array}{c} \omega_{i,t+1}=\left(1-\rho \right)\omega_{i,t}+\rho ,\\ \mu_{i,t+1}=\left(1-\alpha \right)\mu_{i,t}+\alpha M_{t},\\ \delta_{i,t+1}=\left(1-\alpha \right)\delta_{i,t}+\alpha {\left(M_{t}-\mu_{i.t}\right)}^{T}\left(M_{t}-\mu_{i,t}\right),\\ \alpha =\rho g\left(M_{t},\mu_{i.t},\sigma_{i,t}\right), \end{array}$$

where *ρ* is the learning rate of the model, which ranges from 0 to 1, and *α* is the parameter update factor, which determines the speed of the update.

After the update is complete, use the value of *ω*_*i*,*t*_/*δ*_*i*,*t*_ to sort the K Gaussian distributions

(5) $$\begin{array}{c} B=\text{argmin}\left(\sum_{k=1}^{b}\omega_{k}>T\right). \end{array}$$

The effect of background subtraction on the gray-scaled dance video image using the Gaussian mixture model is shown in Figure 2:

### 3.2. Feature Extraction of Dance Images

Optical flow calculation can accurately calculate the changes of dance movements without missing the movement changes of small limbs. The calculation formula is as follows:

(6) $$\begin{array}{c} E\left(w\right)=E_{\text{color}}\left(w\right)+\gamma E_{\text{grad}}\left(w\right)+\alpha E_{\text{smooth}}\left(w\right)+\beta E_{\text{match}}\left(w,w_{1}\right)+E_{\text{desc}}\left(w_{1}\right),\\ E_{\text{color}}\left(w\right)=\int_{\Omega }\Psi \left({\left|I_{2}\left(x+w\left(x\right)\right)-I_{1}\left(x\right)\right|}^{2}\right)\text{dx},\\ E_{\text{grad}}\left(w\right)=\int_{\Omega }\Psi \left({\left|\nabla I_{2}\left(x+w\left(x\right)\right)-\nabla I_{1}\left(x\right)\right|}^{2}\right)\text{dx},\\ E_{\text{smooth}}\left(w\right)=\int_{\Omega }\Psi \left({\left|\nabla \mu \left(x\right){|}^{2}+|\nabla v\left(x\right)\right|}^{2}\right)\text{dx},\\ E_{E}\left(w_{1}\right)=\int \delta \left(x\right){\left|f_{2}\left(x+w_{1}\left(x\right)\right)-f_{1}\left(x\right)\right|}^{2}\text{dx}. \end{array}$$

The audio signal is stored in *y*, the length of *y* is *N*, the sampling rate is *fs*, and the formula for framing is as follows [20]:

(7) $$\begin{array}{c} fs=\frac{\left(N-\text{olap}\right)}{\text{dis}}=\frac{\left(N-\text{wlen}\right)}{\text{dis}+1}. \end{array}$$

Calculate the energy features of audio [21]

(8) $$\begin{array}{c} y_{k}\left(j\right)=\text{win}\left(j\right)\cdot x\left(\left(k-1\right)\cdot \text{dis}+j\right),1\leq j\leq L,1\leq k\leq f,\\ M\left(k\right)=\sum_{j=0}^{L-1}\left|y_{k}\left(j\right)\right|,1\leq k\leq f. \end{array}$$

Among the changing dance moves in a dance video, audio features can extract a representative frame

(9) $$\begin{array}{c} V=\frac{\left|H_{\text{current}}-H_{\text{key}}\right|}{H_{\text{key}}}. \end{array}$$

The similarity matching of human body poses is to realize the measure of the difference or similarity of the poses of different human bodies [19]

(10) $$\begin{array}{c} D=\text{sqrt}\left({\left(x_{1}-x_{2}\right)}^{2}+{\left(y_{1}-y_{2}\right)}^{2}\right),\\ D=\text{sqrt}\left({\left(x_{1}-x_{2}\right)}^{2}+{\left(y_{1}-y_{2}\right)}^{2}+{\left(z_{1}-z_{2}\right)}^{2}\right). \end{array}$$

Stop motion the image in the dance video, and then use the image block marker matrix to calculate the dance motion target, and get

(11) $$\begin{array}{c} L_{IB}\left(m,n\right)=\left\{\begin{array}{cc} 2, & \text{SAD}\left(m,n\right)>t_{\text{SAD}},\\ 1, & \text{IBSCI}\left(m,n\right)>t_{\text{IBSCI}},\\ 0, & \text{else.} \end{array}\right. \end{array}$$

Get the dance action gait contour target [22]

(12) $$\begin{array}{c} Z_{k}\left(x,y\right)=\left\{\begin{array}{cc} 255, & \left|F_{k}\left(x,y\right)-B_{k}\left(x,y\right)\right|\geq \text{Th,}\\ 0, & \text{otherwise.} \end{array}\right. \end{array}$$

## 4. Test Experiments

### 4.1. Simulation Experiment

Human posture can be directly used as feature information for statistical action recognition. The experimental dance collection device is based on the intelligent sensor dance action database, which contains twenty groups of dance action combinations. The music and dance videos include two types of videos: one is a video of a combination of dance movements and the other is to collect data on the combined movements according to the type of movements. The video clip of each dance is about 20 seconds. The test set used in the experiment comes from the dance videos on the Internet. The intelligent sensor music and dance collection mode proposed in the article is compared with the recognition effect of the mechanical motion capture model and the optical motion capture model, and the recognition effect of the feature description is compared with different regions of the human body. The specific experimental data are as follows:

According to the experimental results in Table 2 and Figure 3, we can conclude that in the dance video image extraction process, the feature recognition effect of the algorithm proposed in this article is the highest among the three models. The recognition effect of the upper body is 66.1, the recognition effect of the lower body is 61.0, and the recognition effect of the whole image can reach 73.4. The recognition effect of optical motion capture is the lowest, the recognition effect of the whole image can only reach 60.4, and the recognition effect of mechanical motion capture is in the middle, and the recognition effect of the whole image is 69.1.

According to the data in Table 3 and Figure 4, we can conclude that in the process of statistical experiments on the recognition of different regions of the human body, the recognition effect of the intelligent sensor model proposed in this article is still the highest among the three models, and the recognition effect of the upper body is 33.9, the recognition effect of the lower body is 34.5, and the recognition effect of the whole body is 40.7. The full-body recognition effect of mechanical motion capture is 30.4, and the full-body recognition effect of optical motion capture is 22.4. According to the statistics of the two experimental results, it can also be shown that the recognition effect of the intelligent sensor dance acquisition model proposed in the article is optimal.

### 4.2. Comparative Experiment

In order to verify the effectiveness of the acquisition of music and dance movements by smart sensors on the effect of dance teaching, the experiment chose the method of comparative experiment, and the experiment selected the students who took aerobics as the research object in the 2019 grade of a university. In the experiment, 150 students who took aerobics as an elective were randomly divided into three groups: the routine group, the experimental group, and the training group. Before the experiment, a simple questionnaire survey was conducted on the members of the three groups to understand their learning motivation and learning efficiency. The experimental results showed that the *P* value was greater than 0.05, indicating that there was no significant difference between the three groups of students' learning motivation and learning efficiency. The experiment compares the students' dance performance of traditional music and dance collection methods and smart sensor music and dance collection methods, and observes the superiority of smart sensors in music and dance collection. In order to ensure the objectivity of the experimental data, the three groups of data were tested separately, and the main test contents were movement range, movement strength, movement consistency, movement specification, and 4 parts. The specific experimental data are as follows:

According to the data in Table 4 and Figure 5, we can conclude that under the traditional music and dance collection mode, the dance performance of the training group is the highest, with a range of movements of 80 points, strength of movements 77 points, consistency of movements 75 points, regularity of movements 74 points, and regularity points of 74 points. The dance score of the group was the lowest, with 76 points of movement range, 74 points of movement strength, 72 points of movement coherence, and 70 points of movement standardization. The experimental group's performance was in the middle of the two. In the traditional music and dance collection mode, the *P* values of the four test parts are all greater than 0.05, indicating that under the traditional music and dance collection mode, the differences between the four test modules are not significant.

According to the data in Table 5 and Figure 6, from the analysis of the evaluation results between the conventional group, the experimental group, and the training group, the overall situation of the students in the conventional training group is slightly improved compared with the traditional music and dance collection mode. The *P* values of action coherence are all less than 0.05, indicating that there is a large gap between the three. Among them, the *P* value of action normativeness is 0.05, which has a very significant difference. Compared with the traditional mode, the four test modules of the training group have improved effects. Combined with the evaluation results of the three groups in the traditional music and dance collection mode, we can conclude that under the condition that the initial conditions are basically the same, and the training conditions and environment are basically the same, the trainees who use the smart sensor music and dance collection training method are better in physical fitness. The indicators have been better improved, and the effect is greatly optimized compared with the training effect in the traditional music and dance collection mode.

### 4.3. Model Checking

#### 4.3.1. Evaluation Criteria

The evaluation criteria are shown in Table 6.

#### 4.3.2. Specific Tests

In order to test the performance of the proposed smart sensor-based music and dance acquisition model in music and dance acquisition, the experiment improved the proposed model and ran it on the test set and the hybrid test set with mechanical motion capture and optical motion capture respectively. The test set is used to evaluate the generalization ability of the final model, and the mixed test set tunes the model's hyperparameters and is used to make an initial evaluation of the model's ability. ROC is a model evaluation indicator in the field of machine learning. The larger the ROC value of the classifier, the higher the accuracy rate. The specific experimental data are as follows:

According to the data in Table 7 and Figure 7, we can conclude that the accuracy rate of the dance acquisition model based on the smart sensor algorithm proposed in the article is 88.24%, the accuracy rate can reach 88.96%, the improved accuracy rate can reach 91.46%, and the accuracy rate can reach 91.79%, which is the highest index value among the four models in the experiment. The accuracy rate of the optical motion capture model is 72.21%, which is the lowest among the four models, and the mechanical motion capture model is in the middle state. According to the ROC curves of the four algorithms, we can also see that the ROC curve values of the article and the improved model are very stable, 0.96. The ROC value of the mechanical motion capture model is low, the ROC curve of the optical motion capture model is more tortuous, and the ROC value is also low. The experimental results also show that the performance of the music and dance acquisition model of the smart sensor is the best.

According to the data in Table 8 and Figure 8, we can conclude that after the test set runs, the performance of the four models has decreased to a certain extent, but the smart sensor dance acquisition model proposed in the article has the lowest degree of decline, and the performance after the decline is still highest among the 4 models, with an accuracy of 90.24% before model improvement and 93.16% after improvement. According to the ROC curves of the four algorithms, we can also see that the ROC curve value of the improved system is very stable, no matter in the test set or the mixed test set, the ROC value has been kept at 0.95, the ROC value before the improvement is stable within the range of 0.85–0.95, the ROC curves of the mechanical motion capture model and the optical motion capture model are more tortuous, and the ROC values are also lower. The experimental results further illustrate that the model proposed in this paper has the best performance.

## 5. Conclusion

Relying on intelligent sensor technology, this paper studies the real-time acquisition method of music and dance gestures. The research idea of the article breaks through the traditional research method and provides a new idea for dance acquisition method with information and intelligent technical means. The general idea of the article is to preprocess the collected dance images, including image grayscale and background detection, to extract the character features in the video images. Then use the principle of intelligent sensor to realize the recognition of dance movements. Although some good achievements have been made in dance collection, there are still some deficiencies in some aspects. In the process of collecting dance video data, only one perspective data can be collected, and multiple perspectives cannot be covered. The dance database of this article has a small amount of information and cannot meet the needs of a large number of dance trainers. In the future research work, we should start to solve these problems.

## Figures and Tables

**Figure 1:** The process of acquiring dance gesture data.

**Figure 2:** Background removal result.

**Figure 3:** Feature description recognition effect statistics.

**Figure 4:** Feature recognition statistics of different regions of the human body.

**Figure 5:** Collection statistics of traditional music and dance.

**Figure 6:** Smart sensor music and dance collection statistics.

**Figure 7:** ROC curve under the test set.

**Figure 8:** ROC curve under the mixed test set.

**Table 1:** Classification statistics of motion capture methods.

Capture method	Structure	Advantage	Disadvantage
Mechanical motion capture	Rigid rod attached to the body	Low cost and less restrictive	Movement is restricted, operations are complex, and data processing is complicated
Optical motion capture	High-precision cameras plus data collection points for joints [16]	Low movement restrictions, low cost, and high accuracy	The later data processing is huge, and the signal requirements are high
Electromagnetic motion capture	Electromagnetic generating equipment and receiving equipment	Inexpensive and fast response	More sensitive to the environment
Video motion capture	Camera and image processing device	High cost and low environmental requirements	The image algorithm is responsible, and the implementation is difficult
Acoustic motion capture	Acoustic emission source and receiving processing device [17]	Low price and high environmental adaptability	Poor accuracy and susceptible to interference

**Table 2:** Comparison of recognition effects of feature description.

Body parts	Smart sensor	Mechanical motion capture	Optical motion capture
Upper body	66.1	60.9	52.8
Lower body	61.0	61.6	52.2
Whole body	67.1	55.7	53.3
Whole image	73.4	69.1	60.4

**Table 3:** Feature recognition effects of different regions of the human body.

Body parts	Smart sensor	Mechanical motion capture	Optical motion capture
Upper body	33.9	25.3	10.0
Lower body	34.5	25.8	10.3
Upper body + lower body	45.6	33.3	23.3
Whole body	40.7	30.4	22.4

**Table 4:** Collection methods of traditional music and dance.

Group	Range of motion	Action strength	Continuity of action	Action norm
Regular group	76	74	72	70
Test group	78	76	73	72
Training group	80	77	75	74
Significant P	0.42	0.33	0.39	0.43

**Table 5:** Smart sensor music and dance collection methods.

Group	Range of motion	Action strength	Continuity of action	Action norm
Regular group	86	84	82	79
Test group	88	86	84	83
Training group	92	88	85	85
Significant P	0.42	0.28	0.23	<0.01

**Table 6:** Evaluation criteria table.

	Metrics	Formula
Accuracy	The accuracy measure refers to the ratio of the number of passing passes to all the numbers [23]. The larger the index value, the more accurate the detection result.	Precision=hits_u_/recset_u_
Recall	The recall criterion refers to the ratio of detections to the theoretical maximum hits [24]. The larger the index value, the more accurate the test result.	Recall=hits_u_/testset_u_
F1 measure	The F1 metric can effectively balance the precision and recall by biasing towards the side with a smaller value [25]. The larger the index value, the more accurate the test result.	F1=2 × Precision × Recall/Precision+Recall

**Table 7:** The performance of each model on the test set.

Model	Accuracy (%)	Precision (%)	Recall (%)	F1 score (%)
Smart sensor dance collection model	88.24	88.96	89.30	89.48
Improved dance collection model	91.46	91.79	91.89	91.45
Mechanical motion capture model	84.13	84.43	84.79	85.19
Optical motion capture model	72.21	75.24	75.46	75.12

**Table 8:** The performance of each model on the mixed test set.

Model	Accuracy (%)	Precision (%)	Recall (%)	F1 score (%)
Smart sensor dance collection model	90.24	90.56	90.89	91.24
Improved dance collection model	93.16	93.89	93.78	94.40
Mechanical motion capture model	87.23	87.93	88.12	88.18
Optical motion capture model	75.14	75.24	75.89	7.12

## Data Availability

The experimental data used to support the findings of this study are available from the corresponding author upon request.
